This article has been retracted.

# miR-330-5p suppresses glioblastoma cell proliferation and invasiveness through targeting ITGA5

**DOI:** 10.1042/BSR20170019

**Published:** 2017-06-21

**Authors:** Linsen Feng, Jianhua Ma, Haiming Ji, Yichun Liu, Weixing Hu

**Affiliations:** 1 Department of Neurosurgery, First Affiliated Hospital of Nanjing Medical University, Nanjing, Jiangsu 210029, China; 2 Department of Neurosurgery, Taixing People’s Hospital, Taixing, Jiangsu 225400, China

**Keywords:** glioblastoma (GBM), ITGA5, invasiveness, miR-330-5p, proliferation

## Abstract

The present study intended to investigate the biological effects of miR-330-5p on glioblastoma (GBM) cell proliferation and invasiveness by targeting integrin α5 (ITGA5). The expressions of miR-330-5p and ITGA5 mRNA in GBM cell lines (U87, U251, and U373) and normal brain glial cell line (HEB) were detected using RT-qPCR. Protein expression of ITGA5 was examined using Western blot. The present study used MTT assay, colony formation assay, Transwell assay, wound healing assay, and flow cytometry analysis in order to determine the biological functions of GBM cells (including cell proliferation, invasion, migration, apoptosis, and cell cycle). The present study applied dual-luciferase reporter gene assay to identify the target relationship between miR-330-5p and ITGA5. miR-330-5p was low-expressed in GBM cell lines while ITGA5 was high-expressed compared with HEB. miR-330-5p could directly target ITGA5 as well as suppress its expression in GBM cells. Up-regulation of miR-330-5p and down-regulation of ITGA5 both have an inhibitory effect on cell proliferation, invasion, and migration. Meanwhile, they could also promote GBM cell apoptosis. miR-330-5p could suppress proliferation and invasion of GBM cells through targeting ITGA5.

## Introduction

Glioblastoma (GBM) is one of the most malignant primary brain tumors. It originates in precursors and glial cells within the nervous system, and occurs most frequently in adults [1,2]. GBM is characterized by its extensive intracranial invasion, aggressiveness, and poor prognosis, with an average survival time of no more than 15 months [3]. Currently, the main conventional therapies for GBM include radiotherapy, surgery removal, chemotherapy, and target therapy [3,4]. Although advanced improvements have been made in the therapeutic regimen, the curative effect of conventional treatments for GBM is still very poor [5]. Therefore, a deeper understanding of the mechanisms and potential pathways of the disease is critical for GBM prevention and clinical treatment. There are several current studies proving that microRNAs (miRs or miRNAs) can regulate the expression of both oncogenes and cancer suppressor genes [6,7].

miRNAs are a kind of small, endogenous, non-coding RNA molecule that has less than 24 nucleotides and performs multiple modulated functions such as the negative regulation of various genes [8]. This kind of miRNA can complimentarily bind to the 3′-untranslated region (3′-UTR) of the corresponding target genes, which eventually inhibits the translation of genes at the transcriptional or post-transcriptional level [9,10]. In the last few years, miRNA has been confirmed to play a vital role in biological processes, including the cell cycle proliferation and apoptosis etc. [11]. Moreover, deregulation of miRNA’s expression has been found to be associated with the progression and development of various types of human cancers [12,13]. miR-330, which was first identified by Weber et al. [14], has been verified to be a tumor-suppressant in lung and prostate tumors [15–17]. However, the molecular mechanisms and functions of miR-300-5p in the regulation of GBM malignancies remain unclear.

It is well known that integrin contains a large number of α/β heterodimeric transmembrane adhesion receptors, which can activate different intracellular signaling pathway and thereby regulate the development of tumor cells including cell proliferation, survival rate, and drug resistance [18,19]. Integrin α5 (ITGA5), which belongs to the integrin α chain family, binds predominantly with integrin β1 [20]. Besides, ITGA5 is considered one of the most plentiful proteins within the extracellular matrix (ECM), and function in cell surface adhesion and signaling [21]. Several previous studies have indicated that ITGA5 can operate in certain cancers—including breast cancer, non-small cancer, and gastric cancer—by activating focal adhesion kinase to promote cell adhesion and migration [20,22–24]. For example, Zhang et al. [25] found that ITGA5 can work with miR-31 in affecting cell invasion and metastasis of gastric cancer. Although ITGA5 has been studied in several different malignancies, few researches have been conducted to evaluate its function and expression level in GBM. With this information in mind, we conducted a series of rigorous cellular level experiments to evaluate the connection between miR-300-5p and ITGA5 as well as their effects on GBM.

## Materials and methods

### Cell culture and transfection

We purchased the human GBM cell lines (U87, U251, and U373) and normal brain glial cell lines (HEB) used in the present study from the Institute of Biochemistry and Cell Biology (Chinese Academy of Sciences, Shanghai, China). RPMI 1640 medium (Gibco, Grand Island, NY) containing 10% fetal bovine serum (FBS) was used to incubate the cell lines at 37°C with 5% CO_2_.

Cell transfections involved miR-330-5p mimics, negative control duplex, ITGA5-cDNA, and ITGA5 siRNA (synthesized by GenePharma, Shanghai, China), and were completed with Lipofectamine^TM^ 2000 reagent (Invitrogen, U.S.A.) according to the manufacturer’s instructions. We settled on five groups including: cells without any dispose were designated as control group; cells that were transfected with negative control duplex were designated as NC group; cells transfected with miR-330-5p mimics were designated as miR-mimics group; cells transfected with ITGA5 siRNA were designated as ITGA5 inhibited group (SiITGA5 group); cells transfected with miR-330-5p mimics and ITGA5-cDNA were designated as miR-mimics+ITGA5 group.

### RT-qPCR

We used TRIzol reagent (Invitrogen Corp., CA, U.S.A.) to isolate total RNA from the cells, and a reverse transcription kit (Fermentas, Pittsburgh PA, U.S.A.) as well as PCR reagent (Invitrogen, CA, U.S.A.) to obtain and amplify cDNA. The sequences of primers for qPCR were illustrated in Table 1. RT-qPCR was used to detect the expression levels of miR-330-5p and ITGA5 mRNA, with U6 and GAPDH as internal controls respectively. The relative expression levels were calculated using the 2^–ΔΔ*C*^_T_ method.

**Table 1:** Sequences of primer for qPCR

cDNA	Forward/Reverse	Sequences 5′→3′
miR-330-5p	F	TCTCTGGGCCTGTGTCTTAGGC
ITGA5	F	AGCCTCAGAAGGAGGAGGAC
	R	TTAATGGGGTGATTGGTGGT
U6	F	CGCTTCGGCAGCACATATAC
	R	TTCACGAATTTGCGTGTCAT
GAPDH	F	CCACATCGCTCAGACACCAT
	R	CCAGGCGCCCAATACG

### Western blot

After a 24-h transfection period, we collected proteins from all the cells and measured them using Western blot. The proteins were separated by 10% sodium dodecyl sulfate polyacrylamide gel electrophoresis (SDS/PAGE) and then transferred to polyvinylidene fluoride (PDVF) membranes. The membranes were then blocked with 5% non-fat milk for 2 h at room temperature and subsequently washed with phosphate buffered saline containing Tween-20 (PBST). Then the membranes were incubated with the first antibody (1 ml) for 2 h, washed with PBST, and then incubated at 4°C overnight with the enzyme-marked secondary antibody (1 ml). Membranes were then rinsed four times with PBST so that the ITGA5 proteins could be observed using electrochemical luminescence (ECL), and finally, the relative expression levels could be calculated.

### MTT assay

Cells were transfected for 24 h and then inoculated in a 96-well plate (100 μl/well). MTT assay was conducted five times after inoculation at 12, 24, 48, 72, and 96 h. After each inculcation, there was another 4-h incubation period at 37°C after supplementing 20 μl MTT solution, then the mixture was centrifuged to remove the supernatant and followed by an addition of 150 μl DMSO. A microplate reader (PowerWave340™, BioTek Instruments, Inc., Winooski, U.S.A.) was then used to measure cell absorbency at 570 nm in order to determine cell viability.

### Colony formation assay

Cells in logarithmic growth phase were harvested and plated in culture dishes, each of which contained 200 cells and 10 ml of culture medium. Then the cells were cultured for 2 weeks at 37°C, 5% CO_2_, and 100% humidity. After cultivation, the supernatant was removed and the cells were washed with PBS. Cells were then fixed with 4% paraformaldehyde for 15 min. GIMSA was added to stain the cells for 30 min, then cell colonies were observed and counted under a microscope.

### Transwell assay

Cells were transfected for 48 h, and then were digested with tyrisin and rinsed with PBS. After rinsing, they were suspended in serum-free medium with a concentration of 5 × 10^4^/ml. The suspension was then seeded into the upper chamber, which was coated with 50 mg/l Matrigel (1:8). Dulbecco’s modified eagle medium (DMEM) containing 10% FBS was then added to the lower chamber. After 24 h of incubation, the cells that failed to pass through the membrane were removed, while those that succeeded in invasion were washed twice with PBS and then immobilized with 95% ethanol. Then the cells were stained with hematoxylin for 10 min and counted under a microscope.

### Wound healing assay

Wound healing assay was utilized to evaluate the migration of GBM cells. After the cells had grown to 70% confluence, a 2.5 μl pipette tip was used to make three paralleled wound lines at the middle and both sides of the medium on the single monolayer cells. Photographs were taken at 0 and 24 h after the scratches were made. Then the wound width of each group was observed and measured.

### Flow cytometry analysis

Cell cycle was detected after a 48-h transfection period. Cells were fixed with 70% ethanol at –20°C and then preserved at 4°C overnight. Ethanol was removed after centrifugation and the cells were then washed with PBS. Then 500 μl of PBS containing 50 μg/ml propidium iodide (PI), 100 μg/ml RNaseA, and 0.2% Triton X-100 were added to the cells followed by an incubation period in the dark at 4°C for 30 min. Finally, cell cycle was detected using flow cytometer (BD Biosciences, NJ, U.S.A.) and distribution was analyzed using ModFit LT software (Verity Software House, ME, U.S.A.). Each experiment was repeated three times.

As for cell apoptosis, cells that were transfected for 48 h were stained with Annexin V-FITC and PI using the Apoptosis Detection Kit (R&D Systems, MN, U.S.A.) according to the instructions, and kept in dark at 4°C for 30 min. After that, cell apoptosis was analyzed by flow cytometry.

### Dual-luciferase reporter gene assay

Wild-type 3′-UTR of ITGA5 as well as mutant 3′-UTR of ITGA5 (GenePharm, Shanghai, China) were amplified and ligated into pmirGLO vector (Promega, Madison, U.S.A.) with luciferase gene. These plasmids were sequenced and co-transfected with miR-330-5p mimics or miR-NC in GBM cells. After a 48-h cultivation period, relative luciferase activity was measured using Dual-Luciferase Reporter Assay System (Promega, Mannheim, Germany).

### Statistical analysis

All data were represented as mean ± standard deviation and analyzed using SPSS 21.0 software (SPSS Inc., Chicago, U.S.A.). Differences between groups were determined by *t*-test or nonparametric rank-sum test, and a chi-square test was used for counting data. *P*<0.05 was considered statistically significant.

## Results

### The expression of miR-330-5p and ITGA5 in GBM cells

The expression levels of miR-330-5p in GBM cell lines (U87, U251, and U373) and normal cell line (HEB) were measured using RT-qPCR. The expression of miR-330-5p was remarkably down-regulated in GBM cell lines compared with that in HEB (*P*<0.05, Figure 1A). The expression of ITGA5 mRNA presented the opposite trend; it was significantly overexpressed in GBM cells (*P*<0.05, Figure 1B). Western blot was conducted in order to further confirm this finding and to examine the expression levels of ITGA5 proteins. The results indicated that ITGA5 protein expression was up-regulated in GBM cells, which was exactly consistent with the mRNA expression of ITGA5 (*P*<0.05, Figure 1C). U251 cells were chosen for further experiments because they showed the lowest expression of miR-330-5p and the highest expression of ITGA5 mRNA.

**Figure 1:** The expressions of miR-330-5p and ITGA5 in GBM cells (**A**) The expressions of miR-330-5p in GBM cell lines (U87, U251, and U373) were significantly lower than that in normal cell line (HEB) detected by qRT-PCR. (**B**) The mRNA expressions of ITGA5 in GBM cell lines were obviously higher than that in HEB cells detected by qRT-PCR. (**C**) The protein expression levels of ITGA5 were higher in GBM cell lines than in HEB cells, with GAPDH as internal control. *P<0.05 compared with HEB group.

### miR-330-5p directly targeted ITGA5

We intended to explore whether miR-330-5p could directly target ITGA5, and predicted that miR-330-5p might bind with ITGA5 3′-UTR by TargetScan database (Figure 2A). In order to verify our prediction, we conducted a dual-luciferase reporter gene assay. As presented in Figure 2B, we found that the luciferase activity in ITGA5-wt group decreased dramatically with the presence of miR-330-5p mimic compared with that of NC (*P*<0.05), suggesting that miR-330-5p could directly target ITGA5. In addition, we used RT-qPCR and Western blot to probe into the effect of miR-330-5p on expression levels of ITGA5. We could easily observe that the expressions of ITGA5 decreased significantly at both mRNA and protein levels in cells transfected with miR-330-5p or siRNA-ITGA5 as compared with the NC or control groups separately. The effects of miR-330-5p mimics could be rescued by overexpression of ITGA5 (*P*<0.05, Figure 2C and D). These results suggested that miR-330-5p can suppress the expression of ITGA5 in GBM cells.

**Figure 2:** miR-330-5p directly targeted ITGA5 (**A**) The binding site between mutant or wild-type ITGA5 3′-UTR and miR-330-5p was predicted by TargetScan. (**B**) Luciferase activity in U251 cells co-transfected with miR-330-5p mimics and wild-type ITGA5 3′-UTR was significantly lower than that of NC in ITGA5-wt group. *P<0.05 compared with NC group. (**C**) RT-qPCR results showed that cells transfected with miR-330-5p or siRNA-ITGA5 presented lower ITGA5 mRNA expression. (**D**) Expression levels of ITGA5 protein detected by Western blot suggested that miR-330-5p could suppress the expression of ITGA5. *P<0.05 compared with control group.

### miR-330-5p inhibits GBM cell proliferation and invasiveness

U251 cells were transfected with miR-330-5p mimics, siRNA-ITGA5, and ITGA5-cDNA to determine the effects of miR-330-5p on GBM cell proliferation. Results of the MTT assay were presented in Figure 3A, we observed no notable difference among the five groups within 12 h after transfection (*P*>0.05). However, with the increase in transfection time, the viability of cells in miR-mimics group and SiITGA5 group was lower than the control or NC groups (*P*<0.05). No significant difference was identified between control, NC, and miR-mimics+ITGA5 groups (*P*>0.05). Therefore, we could conclude that overexpression of miR-330-5p and suppression of ITGA5 can reduce cell viability in GBM. As shown in Figure 3B, we observed a decrease in the number of colony formations in mimics and SiITGA5 groups, compared with that in control, NC, and miR-mimics+ITGA5 groups (*P*<0.05).

**Figure 3:** Effects of miR-330-5p and ITGA5 on cell proliferation and invasion of GBM cells (**A**) Relative cell viabilities detected by MTT assay in mimics and SiITGA5 groups were lower than that in control, NC, and miR-mimics+ITGA5 groups, suggesting that overexpression of miR-330-5p or suppression of ITGA5 could both inhibit cell viability. (**B**) The colonies in mimics and SiITGA5 groups were obviously less than that in control, NC, and miR-mimics+ITGA5 groups. (**C** and **D**) There were fewer cells observed in mimics and SiITGA5 groups, which showed that up-regulation of miR-330-5p and down-regulation of ITGA5 could suppress cell invasiveness. (**E** and **F**) Wound healing assay showed the inhibitory effects of up-regulated miR-330-5p and down-regulated ITGA5 on GBM cell migration. *P<0.05 compared with control group.

We also examined the effects of miR-330-5p on cell invasiveness and migration, as shown in Figure 3C–F. The cells that succeeded in invading the membranes in mimics group and SiITGA5 group were significantly less than that in control, NC, and miR-mimics+ITGA5 groups (*P*<0.05, Figure 3C and D). The results of wound healing assay indicated that the migration index of cells in mimics and SiITGA5 groups was apparently lower compared with control, NC, and miR-mimics+ITGA5 groups (*P*<0.05, Figure 3E and F). These results all demonstrated that either up-regulation of miR-330-5p or down-regulation of ITGA5 has an inhibitory effect on cell invasion and migration, whereas overexpression of ITGA5 could antagonize the effects of miR-330-5p mimics.

### Effects of miR-330-5p and ITGA5 on cell cycle and apoptosis of GBM cells

The cell cycle analyzed by flow cytometry indicated that cells in mimics and SiITGA5 groups were mainly arrested in G_0_/G_1_ phase and there were fewer cells in S phase compared with control, NC, and miR-mimics+ITGA5 groups (*P*<0.05, Figure 4A and B). This demonstrated that up-regulation of miR-330-5p or down-regulation of ITGA5 can negatively influence proliferation of GBM cells. Furthermore, we compared the apoptosis rates of U251 cells in different groups. As displayed in Figure 4C and D, the apoptosis ratio was significantly higher in mimics or SiITGA5 group than that in control, NC, and miR-mimics+ITGA5 groups (*P*<0.05). These results suggested that miR-330-5p might act as an inhibitor in GBM cell progress.

**Figure 4:** Effects of miR-330-5p and ITGA5 on cell cycle and apoptosis of GBM cells (**A** and **B**) The cell cycle distribution of U251 cells in different groups showed that cells in mimics or SiITGA5 had higher G_0_/G_1_ phase and lower S phase compared with cells in control, NC, and miR-mimics+ITGA5 groups. (**C** and **D**) The apoptosis rate of U251 cells transfected with miR-330-5p mimics or siRNA-ITGA5 was significantly higher than cells in control, NC, and miR-mimics+ITGA5 groups. *P<0.05 compared with control group.

## Discussion

In recent years, many studies have indicated that abnormal expression of ITGA5 is correlated to local tumor growth and metastasis, and can contribute to cancer invasion and migration [19,20]. Meanwhile, Tréhoux et al. [26] and Mao et al. [27] also found that miR-330 was related to many human cancers including pancreatic cancer, malignant melanoma, and prostate cancer [28]. Although miR-330-5p and ITGA5 have been studied many times before, the relationship between the two modulators and their functional roles in GBM are still unknown. We can conclude from the present study that both up-regulation of miR-330-5p or down-regulation of ITGA5 have an inhibitory effect on cell proliferation and invasion in GBM. Furthermore, there exists a direct targeting relationship between miR-330-5p and ITGA5.

Through cell transfections and a series of functional assays, we discovered that miR-330-5p mimics could inhibit the migration, invasion, and proliferation ability of U251 cell lines. Meanwhile, apoptosis rate was significantly higher in the miR-mimics group, compared with that in control group, which further demonstrated that miR-330-5p could accelerate the apoptosis of GBM cells. Similarly, Li et al. [29] has also found that miR-330 can negatively regulate proliferation and promote apoptosis of colorectal cancer cells, which was consistent with our findings in terms of the effects of miR-330-5p on cancer cell progress. However, there have been several researches that indicate that miR-330 can also act as an oncogenic mRNA with the function of promoting the anti-apoptosis, invasion, migration, and proliferation of human GBM cells [30,31]. The main cause of this contrary result is that certain miRNAs contain many potential targets, and the mechanism differs for each target.

ITGA5 has been widely accepted as involved in the process of invasiveness and tumorigenesis [20,32]. In our research, the expression level of ITGA5 in SiITGA5 group was down-regulated at both mRNA and protein levels, which means that ITGA5 might work as a facilitator in GBM. Migration, invasion, and proliferation ability could be significantly suppressed by knocking out the ITGA5 gene in GBM compared with the NC and control groups. These results were in accordance with the study conducted by Xie et al. [20] who found that ITGA5 could promote growth, migration, and invasion of esophageal squamous cell carcinoma (ESCC) cells. However, we also found that multiple miRNAs (except miR-330-5p) could also target ITGA5, including miR-128, miR-31, miR-26a, and miR-205 [23,25,33,34]. Several other factors could modulate the expression of ITGA5 as well. Hsia et al. [35], for example, found that the absence of matrix-capable fibronectin could result in rapid degradation of ITGA5 by targeting the internalized receptor.

Although we found a novel target relationship between miR-330-5p and ITGA5 in GBM, there are still some limitations in the present study. As mentioned before, we cannot verify that there is no other factor involved in the mechanism of miR-330-5p and ITGA5 in GBM. In addition, all our experiments based on cell level, whether the up-regulation of miR-330-5p or the suppression of ITGA5 would have effects on the progression of GBM patients is still unknown. Therefore, *in vivo* experiments are needed for further investigation.

In conclusion, our study demonstrated that miR-330-5p could act as a tumor suppressor for GBM cells by down-regulating the expressions of ITGA5 in both protein and mRNA levels, and either up-regulated miR-330-5p or down-regulated ITGA5 could reduce cell abilities of proliferation, invasion, and migration while promoting cell apoptosis. Our findings could enhance the understanding of GBM pathogenesis and might provide a new direction for GBM treatment.

## Abbreviations

GBM: glioblastoma
ITGA5: integrin α5
PBST: phosphate buffered saline containing Tween-20
PI: propidium iodide
RT-qPCR: reverse transcription-quantitative polymerase chain reaction
RPMI: roswell Park Memorial Institution
GAPDH: glyceraldehyde-3-phosphate dehydrogenase
